The article "Autophagy in Muscle of Glucose-Infusion Hyperglycemia Rats and Streptozotocin-Induced Hyperglycemia Rats via Selective Activation of m-TOR or FoxO3" was retracted in 2019. Reasons: concerns about the data; concerns about the images; concerns about the results or conclusions.

# Autophagy in Muscle of Glucose-Infusion Hyperglycemia Rats and Streptozotocin-Induced Hyperglycemia Rats via Selective Activation of m-TOR or FoxO3

**DOI:** 10.1371/journal.pone.0087254

**Published:** 2014-02-03

**Authors:** Pengfei Lv, Jian Huang, Jian Yang, Yujie Deng, Jun Xu, Xiaoyan Zhang, Wenyi Li, Hongli Zhang, Ying Yang

**Affiliations:** Department of Endocrine and Metabolic Diseases, Shanghai Institute of Endocrine and Metabolic Diseases, Shanghai Clinical Center for Endocrine and Metabolic Diseases, Ruijin Hospital, Shanghai Jiaotong University School of Medicine, Shanghai, China; Van Andel Institute, United States of America

## Abstract

Autophagy is a conserved process in eukaryotes required for metabolism and is involved in diverse diseases. To investigate autophagy in skeletal muscle under hyperglycemia status, we established two hyperglycemia-rat models that differ in their circulating insulin levels, by glucose infusion and singe high-dose streptozotocin injection. We then detected expression of autophagy related genes with real-time PCR and western blot. We found that under hyperglycemia status induced by glucose-infusion, autophagy was inhibited in rat skeletal muscle, whereas under streptozotocin-induced hyperglycemia status autophagy was enhanced. Meanwhile, hyperglycemic gastrocnemius muscle was more prone to autophagy than soleus muscle. Furthermore, inhibition of autophagy in skeletal muscle in glucose-infusion hyperglycemia rats was mediated by the m-TOR pathway while m-TOR and FoxO3 both contributed to enhancement of autophagy in gastrocnemius muscle in streptozotocin-induced hyperglycemia rats. These data shows that insulin plays a relatively more important role than hyperglycemia in regulating autophagy in hyperglycemia rat muscle through selectively activating the m-TOR or FoxO3 pathway in a fiber-selective manner.

## Introduction

Hyperglycemia impairs cell function and biological processes, leading to severe physical injury and increased mortality [1], [2], [3]. Recent findings have demonstrated that autophagy is involved in diabetes and diabetes complications such as diabetic nephropathy [4], [5], [6], [7], suggesting that autophagy is closely related to hyperglycemia.

Autophagy is an evolutionarily conserved process in eukaryotes that recycles cellular components [8]. It involves numerous autophagy related genes (ATGs) such as Beclin1, Atg5, Atg7, Atg12. The most typical trigger of autophagy is nutrient starvation [7]. Starvation-induced autophagy was observed in many organisms including liver, muscle, heart, pancreas etc. Compared with most other organs, autophagy in skeletal muscle is more sensitive for an obvious longer time of autophagy activation [9]. Autophagy controls muscle mass during catabolic conditions and required for basal myofiber homeostasis [10], [11]. Recently, He C et al. [12] found that autophagy plays a crucial role in glucose homeostasis in mice muscle during excise, suggesting that autophagy is closely to metabolism in skeletal muscle. However, whether loss of homeostasis, such as hyperglycemia, in turn affected autophagy in muscle got less attention. Thus, our interest was aroused to focus on autophagy in skeletal muscle under hyperglycemia status.

The article "Autophagy in Muscle of Glucose-Infusion Hyperglycemia Rats and Streptozotocin-Induced Hyperglycemia Rats via Selective Activation of m-TOR or FoxO3" was retracted in 2019. Reasons: concerns about the data; concerns about the images; concerns about the results or conclusions.

Skeletal muscle contains slow as well as fast twitch muscle fibers exhibiting different proteomics and transcriptomics [13]. Gastrocnemius muscle is composed mainly by fast-twitch muscle fibers and soleus muscle is composed mainly of slow-twitch muscle fibers [14], [15]. A variety of recent reports have indicated that gastrocnemius and soleus differ in many properties [16], [17], [18], and diversity of responses of different skeletal muscles to starvation-induced autophagy has been observed [9]. The AKT signaling pathway plays a crucial role in autophagy in rat skeletal muscle. Downstream of AKT, m-TOR and FoxO3 regulate autophagy under certain circumstances [19]. Activation of the FoxO3 pathway enhances autophagy [20] while the m-TOR pathway plays a negative role in autophagy [21].

In our study, we focus on autophagy in skeletal muscle (gastrocnemius and soleus) under hyperglycemia induced by different mechanisms. Comparing glucose-infusion hyperglycemia rats (GLU-rats) with streptozotocin-induced hyperglycemia rats (STZ-rats), we found that effect on autophagy in these two hyperglycemia rats was opposite. We attribute this to the different insulin levels and provide evidence that the effect is mediated by the mTOR pathway and FoxO3 pathway. In addition, the response differs in the two fiber types studied.

## Results

### Autophagy is Inhibited in Gastrocnemius of GLU-rats

To investigate autophagy under hyperglycemia status in skeletal muscle, we first studied the gastrocnemius of GLU-rats. GLU-rats showed a significant increase in blood glucose (18±4.0 mmol/L) and insulin (11.0±1.5 mmol/L) levels compared with control rats (6.3±1.1 mmol/L, 0.57±0.50 mmol/L) (Figure 1A), implying that the GLU-rats exhibited hyperglycemia with a high insulin level.

**Figure 1:** Autophagy in gastrocnemius is inhibited in Glucose-infusion hyperglycemia rats (GLU-rats). **A:** GLU-rats were treated with 50% glucose via carotid artery infusion for 24 h (2 mg/kg/h). Control rats were treated with an equivalent volume of 0.9% sodium chloride for 24 h. Blood glucose and insulin levels were measured before the rats were killed. **B:** mRNA levels of LC3, Atg5, Atg7, Atg12, BECN1 were detected by RT-PCR in gastrocnemius. **C:** Gastrocnemius lysates were analyzed by Western blot using anti-LC3, anti-Beclin 1, anti-ATG7 and anti-Actin. (*P<0.05, **P<0.01, ***P<0.001).

The article "Autophagy in Muscle of Glucose-Infusion Hyperglycemia Rats and Streptozotocin-Induced Hyperglycemia Rats via Selective Activation of m-TOR or FoxO3" was retracted in 2019. Reasons: concerns about the data; concerns about the images; concerns about the results or conclusions.

Expression of the autophagy-related genes LC3, Atg5, Atg7, Atg12, and BECN1 was analyzed by RT-PCR (Figure 1B). Compared with control rats, mRNA levels of LC3, Atg7, BECN1 significantly decreased while Atg5, Atg12 showed a weak decrease that was not statistically significant. To examine whether translation levels were affected, we used Western blot to detect LC3, Beclin1 and ATG7 (Figure 1C). LC3-II, which is one marker for autophagy [22], was showed a dramatic decrease in GLU-rats. Compared with control rats, Beclin1, an essential autophagy related protein in skeletal muscle, was also significantly reduced. Since the ratio of LC3-II to LC3-I may be more correlated with autophagy than the absolute levels [22], we compared the ratio LC3-II/LC3-I between GLU-rats and control rats (Figure 1C) and also found a significant decrease. Therefore, autophagy was suppressed in gastrocnemius of GLU-rats.

### Autophagy is Enhanced in Gastrocnemius of STZ-rats

Next, we investigated autophagy in gastrocnemius of the other hyperglycemia rat model, STZ-rats, which was established by a single high-dose of streptozotocin and characterized by damage toβcells. In order to eliminate the potential possibility that STZ may directly induce autophagy, we performed western blot in C2C12 muscle fibers and got a negative result (Figure S1).

STZ-rats showed a significant increase in blood glucose level (25±3.0 mmol/L) compared with control rats (6.1±1.5 mmol/L). However, the insulin level in STZ-rats (0.15±0.020 mmol/L) exhibited a dramatic decrease compared with control rats (1.2±0.11 mmol/L), which differed from GLU-rats (Figure 2A).

**Figure 2:** Autophagy in gastrocnemius is triggered in Streptozotocin-induced hyperglycemia rats (STZ-rats). **A:** STZ-rats were treated with streptozotocin via intraperitoneal injection (5 mg/kg). Control animals received an equivalent volume of citric acid buffer. Blood glucose and insulin levels were measured before rats were killed. **B:** RT-PCR was performed to detect the mRNA levels of LC3, Atg5, Atg7, Atg12, and BECN1 in gastrocnemius. **C:** Protein levels of LC3, Beclin1 and ATG7 were analyzed by Western blot in gastrocnemius. (**P<0.01, ***P<0.001).

RT-PCR and western blot showed that the mRNA levels of the autophagy related genes LC3, Atg5 and BECN1 significantly increased, while Atg5 and Atg12 showed a slight increase (Figure 2B). The changes in the levels of the autophagy related proteins mirrored the changes in the mRNAs. The translation levels of LC3-II, Beclin1 and LC3-II/LC3-I showed a statistically significant increase, with ATG7 showing a marginal increase (Figure 2C). Thus, autophagy was enhanced in the gastrocnemius of STZ-rats.

The article "Autophagy in Muscle of Glucose-Infusion Hyperglycemia Rats and Streptozotocin-Induced Hyperglycemia Rats via Selective Activation of m-TOR or FoxO3" was retracted in 2019. Reasons: concerns about the data; concerns about the images; concerns about the results or conclusions.

### Autophagy in the Soleus in the Two Hyperglycemia Rat Models

To investigate whether soleus differs from gastrocnemius in skeletal muscle autophagy under hyperglycemia, the autophagy related proteins LC3, Beclin1, ATG7 were analyzed by western blot in soleus of the two hyperglycemia rat models. In GLU-rats, LC3-II/LC3-I and Beclin1 showed a statistically significant decrease, while ATG7 exhibited a slight decrease (Figure 3A). Although autophagy in the gastrocnemius and soleus of GLU-rats were both reduced, the soleus showed a lesser decrease compared with the gastrocnemius. However, in STZ-rats, expression of the autophagy related proteins LC3, Beclin1 and ATG7 in the soleus remained unchanged compared with control rats (Figure 3B).

**Figure 3:** Autophagy alteration in soleus of GLU-rats and STZ-rats. Soleus lysates were analyzed by Western blot using anti-LC3, anti-Beclin 1, anti-ATG7 and anti-Actin in GLU-rats (**A**) and STZ-rats (**B**) compared with control rats. (*P<0.05).

### M-TOR and FoxO3 are Involved in Autophagy in Skeletal Muscle in Hyperglycemia Rats

From the above results, the two hyperglycemia rat models have nearly opposite effects on autophagy in skeletal muscles. We investigated whether m-TOR and FoxO3 [19] are involved in mediating this process.

P-S6 and p-FoxO3a are commonly used as indicators for activation of the m-TOR pathway and FoxO3 pathway, respectively. In GLU-rats, we observed a noticeable activation of m-TOR in gastrocnemius (Figure 4A) and soleus (Figure 4B), as determined by an increase of p-S6. Meanwhile, the FoxO3 pathway showed no significant alteration in skeletal muscle of GLU-rats. These results indicate that activation of the m-TOR pathway led to the repression of autophagy. In STZ-rats, the alteration in the m-TOR pathway in gastrocnemius was the reverse of that in GLU-rats; p-S6 decreased and p-FoxO3a significantly increased, indicating repression of m-TOR together with activation in FoxO3 led to enhancement in autophagy in the gastrocnemius. In soleus of STZ-rats, no significant alteration in the m-TOR or FoxO3 pathway was detected, in which correlates with no change in autophagy (Figure 4D). The above results suggest that m-TOR is mainly involved in autophagy in hyperglycemia rat skeletal muscle. In addition, FoxO3 is involved in the enhancement of autophagy in the gastrocnemius in STZ-rats. The M-TOR and FoxO3 pathways showed no alteration in the soleus of STZ-rats which may may due to the non-sensitive property to lack of insulin of the soleus fiber in STZ-rats [23]. Alteration in p-mTOR was also detected as shown in supplement materials (Figure S2).

The article "Autophagy in Muscle of Glucose-Infusion Hyperglycemia Rats and Streptozotocin-Induced Hyperglycemia Rats via Selective Activation of m-TOR or FoxO3" was retracted in 2019. Reasons: concerns about the data; concerns about the images; concerns about the results or conclusions.

**Figure 4:** Signaling pathway involved in autophagy in muscle of GLU-rats and STZ-rats. Gastrocnemius lysates (**A**) and soleus lysates (**B**) from GLU-rats were analyzed by Western blot using anti-pS6, anti-pFoxO3 and anti-Actin and compared with control rats. In STZ-rats, western blots were performed with these same antibodies in gastrocnemius (**C**) and soleus (**D**) and compared with control rats. (***P<0.001).

## Discussion

In our study, we found that autophagy was altered in hyperglycemia rat skeletal muscles, and the effects were opposite in the two hyperglycemia models. Autophagy was inhibited in both gastrocnemius and soleus and mediated by the m-TOR pathway in GLU-rats. In STZ-rats, autophagy was enhanced in the gastrocnemius and mediated by the m-TOR and FoxO3 pathway, while autophagy in the soleus was unchanged. In addition, the gastrocnemius was more sensitive to autophagy than the soleus in hyperglycemia rats.

The glucose-infusion hyperglycemia model and the streptozotocin-induced hyperglycemia model are both classic hyperglycemia models that are used widely in research. In the former model, pancreatic β cell proliferation is activated, leading to a relatively higher insulin level [24]. In the latter model, the single high dose of streptozotocin induces damage in rat β cells [25], causing a lower insulin level. The difference in autophagy observed in our study suggested that insulin may be a crucial regulator to autophagy under hyperglycemia conditions. Actually, high fat diet induced hyperinsulinemia was reported to suppress autophagy in mice liver [26]. However, more specific researched are needed to certificate the relationship between insulin and autophagy in skeletal muscle under hyperglycemia.

The gastrocnemius was found to be more sensitive to autophagy than the soleus. The diversity of autophagy responses in skeletal muscle may due to different regulation of protein synthesis and degradation in fast-twitch and slow-twitch muscle fibers [27]. As previously reported, the gastrocnemius is more prone to be affected by external changes such as food deprivation, resulting in protein turnover [27], [28]. Since autophagy is a process of degradation, our observations seems to be consistent with previous studies. However, we didn’t detect specific markers for protein synthesis or degradation in this study. Therefore, although we found that gastrocnemius and soleus differed in responses to autophagy, underlying mechanism needs further evidence. What’s more, different oxidative capacity of fast-switching muscle and slow-switching muscle may be another cause. Fast-switching muscle, which possesses a low oxidative capacity, showed a greater extent in basal and starvation-induced autophagy [29]. In STZ-rats,results were more complicate since we did not detect an alteration in autophagy in the soleus. Different properties of muscle fibers in STZ-rats aroused researchers’ attention ever since 1975. Armstrong R et al pointed out that soleus was not sensitive to lack of insulin induced by STZ, exhibiting a least alteration in histochemical properties. Maybe our results could be a supplement to their research that soleus also appeared to be least affected related to autophagy under hyperglycemia status [23].

The article "Autophagy in Muscle of Glucose-Infusion Hyperglycemia Rats and Streptozotocin-Induced Hyperglycemia Rats via Selective Activation of m-TOR or FoxO3" was retracted in 2019. Reasons: concerns about the data; concerns about the images; concerns about the results or conclusions.

The M-TOR pathway showed detectable changes in the two skeletal muscle in both GLU-rats and STZ-rats, while FoxO3 changed only in gastrocnemius in STZ-rats. Maybe the roles of mTOR and FoxO3 playing in protein turnover was a potent cause. mTOR regulates cell function mainly via regulation of protein synthesis [30] while FoxO3 mainly controls protein degradation [31]. Autophagy is a main pathway of degradation [32]. FoxO3 acted together with m-TOR when autophagy was activated, whereas m-TOR played an important role alone when autophagy was inhibited.

The alteration in autophagy in hyperglycemia rats is shown in Figure 5. In GLU-rats, hyperglycemia associated with a high insulin level activated the m-TOR pathway and inhibited autophagy in the gastrocnemius and soleus. The gastrocnemius is more sensitive to autophagy, so the change in autophagy in the gastrocnemius was more significant than in the soleus. In STZ-rats, hyperglycemia associated with lack of insulin inhibited the m-TOR pathway and activated FoxO3 pathway, triggering autophagy in the gastrocnemius. Our data suggests that insulin may play a relatively more important role than hyperglycemia in autophagy in hyperglycemia rat muscle in a fiber-selective manner, with both mTOR and FoxO3 involved. These findings might provide a new understanding of autophagy under hyperglycemia status in skeletal muscle. However, more research will be needed to specify the underlying mechanism.

**Figure 5:** Autophagy in hyperglycemia rat skeletal muscle. In GLU-rats, the m-TOR pathway is activated in gastrocnemius and soleus, inhibiting autophagy. In STZ-rats, the m-TOR pathway is repressed and the FoxO3 pathway is activated in gastrocnemius, enhancing autophagy.

## Materials and Methods

### Animals

Four-week-old female SD rats (weight = ±200 g) were purchased from SLAC Laboratory Animal Co. Ltd. (Shanghai, China). All animals were housed at 18°C–25°C under 12 h light and dark cycles and allowed access to food and water ad libitum. The National Institutes of Health principles of laboratory animal use and care were strictly followed with institutional approval of Shanghai Institutes of Biological Sciences, Chinese Academy of Sciences.

The article "Autophagy in Muscle of Glucose-Infusion Hyperglycemia Rats and Streptozotocin-Induced Hyperglycemia Rats via Selective Activation of m-TOR or FoxO3" was retracted in 2019. Reasons: concerns about the data; concerns about the images; concerns about the results or conclusions.

### Reagents and Antibodies

RIPA, protease inhibitor, phosphatase inhibitor, and streptozotocin were obtained from Sigma (St. Louis, MO, USA); Trizol was from GIBCO-BRL (Grand Island, NY); SuperScript III, Oligo(dT) were from Invitrogen (Carlsbad, CA, USA); citric acid was from Shanghai Chemical Reagent Limited Company (Shanghai, China); 0.45% Sodium Chloride Injection, 50% Glucose Injection were from Ruijin Hospital (Shanghai, China); RT-PCR detection kit was from Takara (Kyoto,Japan); BCA protein assay kit was from Thermo Scientific (Rockford, IL, USA); Pierce ECL Western blotting substrate was from Thermo Scientific (Rockford, IL, USA). Anti-LC3 was obtained from Sigma (St. Louis, MO, USA); anti-Beclin1, anti-Atg7, anti-pS6 (ser235/236), anti-pFOX03a (ser318/321) were from Cell Signaling Technology (Beverly, MA, USA); anti-Actin was from Abmart (Shanghai, China).

### Development of GLU-rats and STZ-rats

GLU-rats were treated with 50% glucose injection via carotid artery infusion for 24 h (5 g/kg/h, n = 6). Control animals received an equivalent volume of 0.45% sodium chloride (n = 6); STZ-rats were treated with streptozotocin via intraperitoneal injection (65 mg/kg, n = 6). Control animals received an equivalent volume of citric acid buffer (n = 6). Glucose level and insulin level were detected from the second day after streptozotocin injection until rats were killed in the forth day, then gastrocnemius and soleus muscle were prepared for western blot and RT-PCR.

### Western Blotting

Soluble lysates (20 µg per lane) were subjected to 10% or 12% sodium dodecyl sulfate polyacrylamide gel electrophoresis (SDS-PAGE). Proteins were then transferred to nitrocellulose membranes and blocked with 5% nonfat milk/TBST for 1 h at room temperature. Membranes were incubated with primary antibodies (diluted by 1∶1000) for 18 h at 4°C. After washing membranes with TBST three times, membranes were incubated with horseradish-peroxidase-conjugated antibody for 1 h at room temperature followed by three washings. Western blots were developed using Pierce ECL Western blotting substrate and quantified by Quantity One software.

### RT-PCR

RNA was collected with trizol from all rats. Two micrograms of total RNA was used for first-strand cDNA synthesis by using SuperScript II Reverse Transcription Kit. Primers were designed using Primer 5 software. Duplicate PCR was carried out with the intercalating dye SybrGreen. PCR cycles were programmed on an ABI Prism 7000 Sequence Detection System (Applied Biosystems).

The article "Autophagy in Muscle of Glucose-Infusion Hyperglycemia Rats and Streptozotocin-Induced Hyperglycemia Rats via Selective Activation of m-TOR or FoxO3" was retracted in 2019. Reasons: concerns about the data; concerns about the images; concerns about the results or conclusions.

### Statistics

All values are expressed as means ± S.D. Significances of differences among groups were evaluated using unpaired t test. A P value of less than 0.05 was considered statistically significant.

## Supporting Information

Figure S1 **STZ has no effect on autophagy in C2C12 skeletal muscle cells.** Mature C2C12 skeletal muscle cells were exposed to 2.5/5 mM STZ for 0 h, 3 h, 6 h, 9 h, 12 h and 16 h, then western blot was performed to detect autophagy using anti-LC3 and anti-GAPDH.
(TIF)

Figure S2 **Alteration in p-mTOR in muscles of GLU-rats and STZ-rats.** Gastrocnemius lysates and soleus lysates from GLU-rats and STZ-rats were analyzed by Western blot using anti-p-mTOR and anti-Actin.
(TIF)

## References

[1] QueisserMA, YaoD, GeislerS, HammesH-P, LochnitG, et al (2010) Hyperglycemia impairs proteasome function by methylglyoxal. Diabetes 59: 670–678.2000908810.2337/db08-1565PMC2828656

[2] UmpierrezGE, IsaacsSD, BazarganN, YouX, ThalerLM, et al (2002) Hyperglycemia: an independent marker of in-hospital mortality in patients with undiagnosed diabetes. Journal of Clinical Endocrinology & Metabolism 87: 978–982.1188914710.1210/jcem.87.3.8341

[3] YaoD, BrownleeM (2010) Hyperglycemia-induced reactive oxygen species increase expression of the receptor for advanced glycation end products (RAGE) and RAGE ligands. Diabetes 59: 249–255.1983389710.2337/db09-0801PMC2797929

[4] KumeS, ThomasMC, KoyaD (2012) Nutrient sensing, autophagy, and diabetic nephropathy. Diabetes 61: 23–29.2218737110.2337/db11-0555PMC3237646

[5] ChenZ-f, LiY-B, HanJ-y, WangJ, YinJ-J, et al (2011) The double-edged effect of autophagy in pancreatic beta cells and diabetes. Autophagy 7: 12–16.2093550510.4161/auto.7.1.13607PMC3039729

[6] GonzalezCD, LeeM-S, MarchettiP, PietropaoloM, TownsR, et al (2011) The emerging role of autophagy in the pathophysiology of diabetes mellitus. Autophagy 7: 2–11.2093551610.4161/auto.7.1.13044PMC3359481

[7] RabinowitzJD, WhiteE (2010) Autophagy and metabolism. Science 330: 1344–1348.2112724510.1126/science.1193497PMC3010857

[8] MeijerAJ, CodognoP (2008) Autophagy: a sweet process in diabetes. Cell Metab 8: 275–276.1884035510.1016/j.cmet.2008.09.001

[9] MizushimaN, YamamotoA, MatsuiM, YoshimoriT, OhsumiY (2004) In vivo analysis of autophagy in response to nutrient starvation using transgenic mice expressing a fluorescent autophagosome marker. Molecular biology of the cell 15: 1101–1111.1469905810.1091/mbc.E03-09-0704PMC363084

[10] SandriM (2010) Autophagy in skeletal muscle. FEBS letters 584: 1411–1416.2013281910.1016/j.febslet.2010.01.056

The article "Autophagy in Muscle of Glucose-Infusion Hyperglycemia Rats and Streptozotocin-Induced Hyperglycemia Rats via Selective Activation of m-TOR or FoxO3" was retracted in 2019. Reasons: concerns about the data; concerns about the images; concerns about the results or conclusions.

[11] MasieroE, AgateaL, MammucariC, BlaauwB, LoroE, et al (2009) Autophagy is required to maintain muscle mass. Cell Metab 10: 507–515.1994540810.1016/j.cmet.2009.10.008

[12] HeC, BassikMC, MoresiV, SunK, WeiY, et al (2012) Exercise-induced BCL2-regulated autophagy is required for muscle glucose homeostasis. Nature 481: 511–515.2225850510.1038/nature10758PMC3518436

[13] Drexler HC, Ruhs A, Konzer A, Mendler L, Bruckskotten M, et al.. (2012) On marathons and Sprints: an integrated quantitative proteomics and transcriptomics analysis of differences between slow and fast muscle fibers. Mol Cell Proteomics 11: M111 010801.10.1074/mcp.M111.010801PMC343392722210690

[14] SteinJM, PadykulaHA (1962) Histochemical classification of individual skeletal muscle fibers of the rat. Am J Anat 110: 103–123.1391663110.1002/aja.1001100203

[15] VandervoortA, McComasA (1983) A comparison of the contractile properties of the human gastrocnemius and soleus muscles. European journal of applied physiology and occupational physiology 51: 435–440.668504110.1007/BF00429079

[16] YuanY, ShiX-e, LiuY-g, YangG-s (2011) FoxO1 regulates muscle fiber-type specification and inhibits calcineurin signaling during C2C12 myoblast differentiation. Molecular and cellular biochemistry 348: 77–87.2108003710.1007/s11010-010-0640-1

[17] CanepariM, PellegrinoM, D’AntonaG, BottinelliR (2010) Skeletal muscle fibre diversity and the underlying mechanisms. Acta Physiologica 199: 465–476.2034541510.1111/j.1748-1716.2010.02118.x

[18] GelfiC, VassoM, CerretelliP (2011) Diversity of human skeletal muscle in health and disease: contribution of proteomics. Journal of proteomics 74: 774–795.2141442810.1016/j.jprot.2011.02.028

[19] MammucariC, SchiaffinoS, SandriM (2008) Downstream of Akt: FoxO3 and mTOR in the regulation of autophagy in skeletal muscle. Autophagy 4: 524–526.1836786810.4161/auto.5905

[20] SanchezAM, CsibiA, RaibonA, CornilleK, GayS, et al (2012) AMPK promotes skeletal muscle autophagy through activation of forkhead FoxO3a and interaction with Ulk1. J Cell Biochem 113: 695–710.2200626910.1002/jcb.23399

[21] JungCH, RoS-H, CaoJ, OttoNM, KimD-H (2010) mTOR regulation of autophagy. FEBS letters 584: 1287–1295.2008311410.1016/j.febslet.2010.01.017PMC2846630

[22] KlionskyDJ, AbdallaFC, AbeliovichH, AbrahamRT, Acevedo-ArozenaA, et al (2012) Guidelines for the use and interpretation of assays for monitoring autophagy. Autophagy 8: 445–544.2296649010.4161/auto.19496PMC3404883

[23] ArmstrongR, GollnickP, IanuzzoC (1975) Histochemical properties of skeletal muscle fibers in streptozotocin-diabetic rats. Cell and tissue research 162: 387–393.12680610.1007/BF00220185

The article "Autophagy in Muscle of Glucose-Infusion Hyperglycemia Rats and Streptozotocin-Induced Hyperglycemia Rats via Selective Activation of m-TOR or FoxO3" was retracted in 2019. Reasons: concerns about the data; concerns about the images; concerns about the results or conclusions.

[24] ZhangH, LiW, WangQ, WangX, LiF, et al (2012) Glucose-Mediated Repression of Menin Promotes Pancreatic β-Cell Proliferation. Endocrinology 153: 602–611.2216697510.1210/en.2011-1460

[25] WilsonGL, PattonNJ, McCordJM, MullinsDW, MossmanBT (1984) Mechanisms of streptozotocin- and alloxan-induced damage in rat B cells. Diabetologia 27: 587–591.624157410.1007/BF00276973

[26] LiuH-Y, HanJ, CaoSY, HongT, ZhuoD, et al (2009) Hepatic Autophagy Is Suppressed in the Presence of Insulin Resistance and Hyperinsulinemia INHIBITION OF FoxO1-DEPENDENT EXPRESSION OF KEY AUTOPHAGY GENES BY INSULIN. Journal of Biological Chemistry 284: 31484–31492.1975899110.1074/jbc.M109.033936PMC2781544

[27] VaryTC, KimballSR (1992) Sepsis-induced changes in protein synthesis: differential effects on fast-and slow-twitch muscles. American Journal of Physiology-Cell Physiology 262: C1513–C1519.10.1152/ajpcell.1992.262.6.C15131377447

[28] LiJB, GoldbergAL (1976) Effects of food deprivation on protein synthesis and degradation in rat skeletal muscles. American Journal of Physiology–Legacy Content 231: 441–448.10.1152/ajplegacy.1976.231.2.441961895

[29] Mofarrahi M, Guo Y, Haspel JA, Choi AM, Davis EC, et al.. (2013) Autophagic flux and oxidative capacity of skeletal muscles during acute starvation. Autophagy 9.10.4161/auto.2595523955121

[30] HayN, SonenbergN (2004) Upstream and downstream of mTOR. Genes & development 18: 1926–1945.1531402010.1101/gad.1212704

[31] ZhaoJ, BraultJJ, SchildA, CaoP, SandriM, et al (2007) FoxO3 coordinately activates protein degradation by the autophagic/lysosomal and proteasomal pathways in atrophying muscle cells. Cell metabolism 6: 472–483.1805431610.1016/j.cmet.2007.11.004

[32] KlionskyDJ, EmrSD (2000) Autophagy as a regulated pathway of cellular degradation. Science 290: 1717–1721.1109940410.1126/science.290.5497.1717PMC2732363

